# Treatment of Elderly Femoral Intertrochanteric Fracture by InterTan Intramedullary Nail and PFNA

This article has been retracted.

**DOI:** 10.1155/2022/5020960

**Published:** 2022-07-31

**Authors:** Zhengbing Su, Minghui Yang, Gang Luo, Linlin Liang, Yong Hao

**Affiliations:** ^1^Department of Orthopedics, The Second Affiliated Hospital of Army Medical University, Chongqing 400037, China; ^2^Department of Clinical Laboratory, The Second People's Hospital in Jiulongpo District Chongqing, Chongqing 400000, China

## Abstract

To analyze the treatment of elderly femoral intertrochanteric fracture (EFIF) using InterTan intramedullary nail (InterTanIN) and proximal femoral nail antirotation (PFNA). A total of 75 patients suffering from EFIF receiving intramedullary fixation were retrospectively collected. According to intramedullary fixation methods, the patients were separated into InterTanIN group and PFNA group. Parameters including the surgery time, blood loss, number of X-ray fluoroscopy, hospital stays, bone-healing time, postoperative Harris hip score (HIS) (1 month, 3 months, 6 months, and 12 months), and complications were collected and analyzed. The results showed surgery time, blood loss, and number of X-ray fluoroscopy in InterTanIN group were higher than those in PFNA group (*P* < 0.05). The mean hospital stay in the InterTanIN group was comparable to that in the PFNA group (*P* > 0.05). There was no significant difference in bone-healing time between the InterTanIN group and PFNA group (*P* > 0.05). The postoperative HIS of InterTanIN group was statistically better than PFNA group at the 3rd month and the 6th month (*P* < 0.05). With the extension of recovery time, the gap between the two groups gradually narrowed. The postoperative implant displacement happened more often in the PFNA group than in the InterTanIN group. EFIF treated with InterTanIN or PFNA could achieve good long-term efficacy. Although InterTanIN has the disadvantages of increased operative time, blood loss, and radiation exposure compared to PFNA, the postoperative hip function recovery of InterTanIN seems to be more reliable and stable than PFNA.

## 1. Introduction

Elderly femoral intertrochanteric fracture (EFIF) is a common clinical fracture, which mainly occurs in the population over 60 years. As the aging population increases, the occurrence rate of EFIF increases year-by-year [1]. For the elderly, especially elderly women, traumatic falls are the main pathogenic cause for EFIF. EFIF is also closely related to osteoporosis and bone fragility caused by various factors [2]. Due to the advantages of early rehabilitation and mobility, surgical treatment is the first choice for treating EFIF [3]. Surgical treatment generally includes intramedullary fixation and extramedullary fixation. Compared with extramedullary fixation, intramedullary fixation shows more advantages [4]. It is reported that intramedullary fixation costs less surgery time and causes less blood loss [5–7]. From a biomechanical point of view, intramedullary fixation can effectively share the load of the fracture site. Main nails of intramedullary fixation is closer to the load-bearing axis than extramedullary fixation, which is in line with biomechanical design of the human body. In addition, femoral neck collapse can be reduced in intramedullary fixation because the cortical bone at the proximal end of the fracture is adjacent to the screw [8].

At present, the widely applied intramedullary fixation systems mainly include proximal femoral nail antirotation (PFNA) and InterTan intramedullary nail (InterTanIN). The design of the spiral blade in PFNA can not only compress the cancellous bone to avoid bone loss but also increase the contact area with the bone resulting in enhanced stability and antirotation performance. InterTanIN is a new generation of intramedullary nails designed for proximal femoral fractures. The main nail of InterTanIN has a proximal trapezoidal cross section, which can effectively increase the intramedullary contact area and improve stability. The design of combined interlocking nail in InterTanIN effectively avoids the *Z*-effect of the traditional double nail device. Some researchers recommend the use of PFNA due to its less surgery time, less blood loss, and less hospital stays [9]. However, some researchers believe that InterTanIN has a higher Harris hip score (HIS) and stability [10]. There is still a lot of controversies about the choice of the two intramedullary fixation systems in the treatment of EFIF.

In this study, a total of 75 patients with femoral intertrochanteric fracture were retrospectively collected, and both the intraoperative parameters and postoperative parameters were compared between the InterTan group and PFNA group.

## 2. Materials and Methods

### 2.1. Study Population and Inclusion/Exclusion Criteria

The information about 75 EFIF cases treated with InterTanIN or PFNA from January 2018 to June 2021 were retrospectively collected. Based on intramedullary fixation methods, they were divided into the InterTanIN group including 41 cases and the PFNA group including 34 cases. The flowchart of this study is shown in Figure 1. This research was approved by the ethics committee of our hospital. All patients signed written informed consent before surgery.

#### 2.1.1. Inclusion Criteria

① Age ≥60 years old, follow-up time ≥12 months, complete follow-up data
② The diagnosis of pure EFIF was confirmed by physical examination and imaging examination (X-ray film and CT)
③ In line with the indications for intramedullary fixation, InterTanIN or PFNA was applied for EFIF treatment
④ The operation time should not exceed 1 week after injury

#### 2.1.2. Exclusion Criteria

① Multiple fractures or open fractures caused by violent injury
② Pathological fractures
③ Combined with severe chronic circulatory and respiratory diseases

### 2.2. Surgical Methods

General anesthesia or epidural anesthesia was applied according to the patient's condition and wishes. The lower extremity of patients was immobilized by a traction frame. In order to facilitate intraoperative fluoroscopy, the contralateral limb was in abduction, knee flexion, and hip flexion position. Appropriate traction or various tools were used for closed reduction of the affected limb first. Fluoroscopy was applied to confirm satisfactory reduction.

InterTanIN group: an incision about 4 cm was performed along the outer side of the top of the greater trochanter. After the greater trochanter was exposed, the guide nail was inserted into the medullary cavity and confirmed by fluoroscopy. Selective reaming was performed according to the preoperative and intraoperative evaluation of the medullary cavity. Then, the InterTanIN of appropriate diameter was inserted into the medullary cavity. Two lag screw guide nails were inserted in the direction of the femoral neck through an external guide. After determining the length of the required lag screws by measurement, the lag screws were inserted along the guide nails and confirmed by fluoroscopy. The guide nail was pulled out after confirming satisfactory positions of anterior and lateral. The proximal femur was fixed with interlocking pressure. Then, the distal nail was inserted with guidance.

PFNA group: an incision about 4 cm was performed along the outer side of the top of the greater trochanter, exposing greater trochanter. The guide nail was inserted into the medullary cavity and confirmed by fluoroscopy. Selective reaming was performed according to the preoperative and intraoperative medullary cavity evaluation. Then, PFNA of appropriate diameter was inserted into the medullary cavity. The guide nail was inserted in the direction of the neck. After confirming the position of the guide nail, a spiral blade was inserted along the direction of the guide nail. After confirming the satisfactory position by fluoroscopy, the nails were fixed. Then, the distal nail was inserted with guidance.

Intramedullary nail implantation criteria [11]: the screw blade or lag screw was located in the middle and lower 1/3 of the femoral neck on the anteroposterior radiograph and in the center of the femoral neck on the lateral radiograph; the depth of the helical blade or lag screw could reach the femoral neck. Subchondral bone: tip-apex distance <25 mm. All operations were performed by the same doctor.

### 2.3. Postoperative Treatment

Prophylactic anti-infective therapy was routinely given after operation. Symptomatic treatment was also applied to avoid venous thrombosis according to the VTE score. The patients were instructed to exercise the quadriceps femoris and dorsiflexion of the ankle joint in the early stage and properly flex the knee and hip.

### 2.4. Method of Assessment

The surgery time, blood loss, times of X-ray fluoroscopy, hospital stays, and complications were analyzed in the InterTanIN group and PFNA group. On the first day after the operation, the X-rays were used to examine the reduction and tip-apex distance.

Outpatient follow-up was performed at 1st, 3rd, 6th, and 12th month after the operation. X-rays were taken each time to examine the healing, and HIS was calculated at the same time.

### 2.5. Statistical Analysis

Statistical analysis was performed by SPSS 24.0 (IBM Corp, USA). Measurement data between the InterTanIN group and PFNA group were compared by independent two-sample *t*-test. The count data were compared by chi-square test or Fisher's exact test. *P* < 0.05 was considered statistically significant.

## 3. Results

### 3.1. Subjects

A total of 75 cases were included, as shown in Table 1. No significant difference was observed in gender composition, age, fracture site, AO type, anesthesia method, fracture reduction, and apex distance between the InterTanIN group and PFNA group.

### 3.2. Hospitalization

The average surgery time and blood loss using InterTanIN as shown in Figure 2 were 72.44 ± 11.64 min and 217.3 ± 54.1 ml, respectively, which were statistically higher than those in the PFNA group (64.47 ± 12.63 min and 156.4 ± 50.90 ml, *P* < 0.05). In terms of intraoperative X-ray fluoroscopy, the InterTanIN group (21.39 ± 6.12) also had significantly more fluoroscopy times than the PFNA group (15.53 ± 5.67) (*P* < 0.001). However, no obvious difference was observed in hospital stays in the InterTanIN group (11.71 ± 3.11) and PFNA group (12.03 ± 4.43) (*P* > 0.05).

### 3.3. Complications

Complications generally involved infection, deep vein thrombosis, implant displacement, and secondary surgery, as shown in Table 2. There were 4 cases and 3 cases of wound infection in the InterTanIN group and PFNA group, respectively, which were improved after anti-infection medication and wound dressing care. There were 2 cases and 1 case of deep vein thrombosis in the InterTanIN group and PFNA group, respectively. Notably, 3 patients in the PFNA group developed partial displacement of the implant during follow-up.

### 3.4. Imaging Changes of the Fracture Site

Figures 3 and 4 show the radiographic changes of the fracture site in the InterTanIN group and PFNA group, respectively.

### 3.5. Healing Time

Average healing time of the InterTanIN group and PFNA group as shown in Figure 5 was 12.54 ± 3.81 weeks and 12.94 ± 3.17 weeks, respectively. No obvious difference was observed between the InterTanIN group and PFNA group (*P* > 0.05).

### 3.6. Ipsilateral HIS

Table 3 shows that there was no obvious difference in HIS between InterTanIN thgroup and PFNA group at 1st and 12th month after operation (*P* > 0.05). e HIS in InterTanIN group as shown in Figure 6 was higher than that in the PFNA group at the 3rd and 6th month after surgery (*P* < 0.05), but difference between the two was gradually narrowing.

## 4. Discussion

InterTanIN and PFNA are commonly used intramedullary fixation systems. The operating principles of the two intramedullary fixation devices are similar. The main nails are both anatomically designed. The main difference is that InterTanIN uses a combined interlocking double nail mode, while PFNA uses a helical blade for antirotation and stable support. Both intramedullary fixation devices have pros and cons. The helical blade implantation of PFNA is more convenient than the double nail implantation of InterTanIN, but the ability to stabilize the fracture end in PFNA may not be as good as that in InterTanIN. Biomechanical studies found that InterTanIN had better resistance to varus deformation, femoral head rotation, and inversion than PFNA in simulation experiment performed on femoral specimens [12]. However, whether the biomechanical advantages found in simulation experiment could work in clinical practice is still controversial.

The results of this study showed that the PFNA group had obvious advantages in terms of surgery time, blood loss, and fluoroscopy, which were in line with the findings of the previous research by Zhang et al. [9]. This may be due to the lower difficulty of PFNA. No obvious difference of healing time was observed in the InterTanIN group and PFNA group, which suggested that the fracture healing was not significantly related to the type of implant when the fracture end was well reduced and fixed. Postoperative hip function recovery is the focus of surgical treatment. The hip joint function of the InterTanIN group and PFNA group recovered well at the first month after operation. HIS improved with the increasing of follow-up time. HIS of the InterTanIN group was obviously higher than the PFNA group at the 3rd and 6th month, which may be due to the lower scores of 3 patients with mild displacement of the internal fixation in PFNA group. Although the slight displacement of the helical blade did not cause obvious adverse consequences after proper braking and symptomatic treatment of osteogenesis, it still had a negative impact on the functional recovery of the affected hip joint. At the 12th month after surgery, hip joint function in the InterTanIN group and PFNA group was further recovered, and the difference between the two groups was significantly reduced. Different from this study, some researchers found that no obvious difference in walking ability and HIS was observed in the two groups [9]. The study by Wang et al. showed that InterTanIN was more reliable than PFNA in comminuted and complex EFIF, with significantly fewer intraoperative complications [13]. Zhang et al. retrospectively compared the results of surgical treatment of 174 patients with InterTanIN and PFNA and found that the postoperative HIS of InterTanIN was obviously higher than that of PFNA [10]. In addition, Zhang et al. also found that, at the 18th month after surgery, the HIS even showed a downward trend in the two groups [10]. However, it is worth noting that most of the previous studies were performed in small-sample and retrospective studies, which still needs to be further verified by further randomizedly controlled and multicenter clinical trials with large samples. In addition, small differences in HIS, even if statistically significant, do not fully represent actual differences in postoperative joint function and life quality. Therefore, according to the current evidence, it cannot be determined which intramedullary fixation systems can achieve better quality of life.

The occurrence of complications is an important factor affecting the treatment effect. Complications in this study included wound infection, deep vein thrombosis, and implant displacement. In the PFNA group, except for 3 patients whose implants were slightly displaced and affected the recovery of limb function, complications in the remaining cases were properly managed in a timely manner, and there was no significant effect on the patient's postoperative recovery. Different from this study, many researchers found that the incidence of complications such as leg pain, screw cutout, internal fixation failure, and coxa varus deformity was statistically lower in the InterTanIN group than in the PFNA group [14–16]. In addition, some researchers found that there was great uncertainty on the impact on complications using different internal fixation systems, which might be caused by a small sample group and potential selection bias [17].

## 5. Strengths and Limitations

In this study, there were no significant differences in gender composition, age, fracture site, AO type, anesthesia method, reduction results, and tip-apex distance between the InterTanIN group and PFNA group, which suggests the evaluation parameters of two groups were well comparable. In addition, intraoperative parameters, postoperative parameters, and follow-up parameters were all collected, which could make a more comprehensive evaluation of these two groups and improve the reliability of the results.

There are still some limitations of this study. First, the case numbers included in this research is relatively small, and the follow-up period is not long enough. The reliability of the research conclusions still needs to be verified by further larger-scale prospective randomized experiments. Secondly, the subjects of this study were all cases with relatively complete follow-up data, which might cause a certain selection bias. Some patients with poor curative effect and low follow-up willingness might be excluded from the scope of analysis. Finally, since the selection of cases had a certain time span, changes in the operator's experience might also have a certain impact on the surgical effect.

## 6. Conclusion

All in all, InterTanIN and PFNA can achieve good results in the treatment of EFIF. Although InterTanIN has disadvantages such as longer operation time, intraoperative bleeding, and increased X-ray frequency when used for the treatment of EFIF, the postoperative hip function recovery of InterTanIN may be more stable than PFNA. There is no significant long-term effect between the two intramedullary fixation systems. In actual clinical work, a more suitable internal fixation method should be selected according to the patient's own characteristics.

## Figures and Tables

**Figure 1:** Flow diagram demonstrating methods for the studies.

**Figure 2:** Perioperative variables: (a) hospital stay; (b) no. of fluoroscopy; (c) blood loss; (d) operation time. Note: ^*∗*^*P* < 0.05, ^*∗∗*^*P* < 0.01, and ^*∗∗∗*^*P* < 0.001.

**Figure 3:** The anteroposterior femur X-ray of patient treated with interTanIN. (a) Preoperative anteroposterior femur; (b) postoperative anteroposterior femur; and (c) anteroposterior femur at 12th month after operation.

**Figure 4:** The anteroposterior femur X-ray of patient treated with PFNA. (a) Preoperative anteroposterior femur; (b) postoperative anteroposterior femur; and (c) anteroposterior femur at 12th month after operation.

**Figure 5:** Bone-healing time of patients in the InterTanIN group and PFNA group.

**Figure 6:** HIS of patients in the InterTanIN group and PFNA group.

**Table 1:** EFIF patient demographics.

Factor	InterTanIN group (*n* = 41)	PFNA group (*n* = 34)	*t*/*X*^2^ value	*P* value
Gender				
Male	13 (31.71)	11 (32.35)	0.004	0.952
Female	28 (68.29)	23 (67.65)		

Age (mean ± SD, y)	68.61 ± 6.7	66.97 ± 4.79	1.194	0.236

Side of fracture				
Left	17 (41.46)	15 (44.12)	0.054	0.817
Right	24 (58.54)	19 (55.88)		

AO fracture type, no.				
A2.1	12 (29.27)	7 (20.59)	3.307	0.653
A2.2	15 (36.59)	11 (32.35)		
A2.3	10 (24.39)	14 (41.18)		
A3.1	1 (2.44)	1 (2.94)		
A3.2	2 (4.88)	1 (2.94)		
A3.3	1 (2.44)	0		

Anesthesia, no.				
General	11 (26.83)	7 (20.59)	0.397	0.529
Spinal	30 (73.17)	27 (79.41)		

Reduction results, no.				
Anatomical	34 (82.93)	29 (85.29)	0.078	0.781
Acceptable	7 (17.07)	5 (14.71)		
Poor	0	0		
Tip-apex distance (mm)	22.63 ± 0.96	22.86 ± 1.2	0.937	0.352

**Table 2:** Postoperative complications *n* (%).

Factor	InterTanIN group (*n* = 41)	PFNA group (*n* = 34)
Total	6 (14.63)	7 (20.59)
Wound infection	4 (9.76)	3 (8.82)
Deep venous thrombosis	2 (4.88)	1 (2.94)
Migration of implants	0	3 (8.82)
Reoperation	0	0

**Table 3:** HIS of patients in the InterTanIN group and PFNA group (mean ± SD).

HIS	InterTanIN group	PFNA group	*t* value	*P* value
1st month	74.29 ± 6.78	73.5 ± 5.76	0.519	0.605
3rd month	83.73 ± 5.76	79.82 ± 4.64	3.188	0.002
6th month	83.93 ± 5.98	80.44 ± 6.08	2.494	0.015
12th month	85.29 ± 11	83.18 ± 8.1	0.932	0.355

## Data Availability

The simulation experiment data used to support the findings of this study are available from the corresponding author upon request.
